RETRACTED

# Inhibition of SphK1/S1P Signaling Pathway Alleviates Fibrosis and Inflammation of Rat Myocardium after Myocardial Infarction

**DOI:** 10.1155/2022/5985375

**Published:** 2022-07-13

**Authors:** Xiaokui Wu, Junwei Xu, Xiangyu Li, Jian Dai, Linlin Wang

**Affiliations:** Department of Cardiology, The Affiliated Brain Hospital of Nanjing Medical University, Nanjing Chest Hospital, Nanjing, China

## Abstract

**Objective:**

The sphingosine kinase 1 (SphK1)/sphingosine-1-phosphate (S1P) signaling pathway is involved in fibrosis and inflammatory responses of myocardial tissue after myocardial infarction (MI). The purpose of our study was to explore the role of SphK1/S1P signaling pathway in myocardial injury after MI.

**Materials and Methods:**

We used Sprague-Dawley (SD) rats to make MI models and detected the changes of SphK1 and S1P in rats at 1, 7, and 14 days after MI. SphK1 inhibitor PF543 was used to treat MI rats, and we detected the changes in myocardial function and structure in rats by cardiac function test, 2,3,5-triphenyl tetrazolium staining, and histological staining. In addition, we used H_2_O_2_ to induce H9c2 cell injury to investigate the effect of PF543 on the viability of myocardial cells.

**Results:**

Myocardial tissue lesions and fibrosis were observed at 7 and 14 days after MI, and the expressions of SphK1 and S1P in the injured myocardial tissues increased significantly in day 7 and day 14 in comparison to the control group. After treatment of MI rats with PF543, the structure of rat myocardial tissue was significantly improved and the degree of fibrosis was reduced. After MI, the expression of *α*-SMA and collagen I in the myocardium of rats was significantly increased while PF543 decreased their expression. PF543 also improved the cardiac function of MI rats and reduced the expression of IL-1*β*, IL-6, and TNF-*α* in the serum. PF543 also increased the viability of H9c2 cells *in vitro*.

**Conclusions:**

The inhibition of the SphK1/S1P signaling pathway contributed to the relief of myocardial injury in MI rats. PF543 improved the myocardial structure and function of MI rats and reduced the level of fibrosis and inflammation in MI rats.

## 1. Introduction

Coronary heart disease is a leading cause of death, killing more than 360,000 people every year.

Myocardial infarction (MI) is caused by acute coronary occlusion and leads to myocardial injury in the corresponding blood supply area [1]. Acute MI still frequently leads to heart failure and contributes to cardiovascular morbidity and mortality. Timely restoration of ischemic myocardial blood flow, limitation of infarct size, and improvement of myocardial function have become the standard treatment for MI patients. However, myocardial cells are nonregenerating cells and irreversible injury occurs immediately after 20 minutes of complete ischemia and hypoxia [2]. In addition, during the process of restoring blood supply, the myocardium may also suffer from reperfusion injury, resulting in excessive inflammation and oxidative stress, thereby exacerbating the damage to the myocardial cells [3]. In the repair process after MI, scars formed by fibrous connective tissue without systolic or diastolic function replaced the dead myocardial cells, causing myocardial injury after MI, mainly manifested as cardiac fibrosis and cardiac dysfunction [4]. Therefore, improving myocardial cell viability and reducing the number of dead myocardial cells under ischemic and hypoxic conditions is essential for reducing myocardial injury after MI.

RETRACTED

Sphingosine (Sph) kinase 1 (SphK1) and sphingolipid metabolites are important signaling molecules [5]. SphK1 is an enzyme in the sphingomyelin metabolism pathway, which can convert Sph into sphingosine-1-phosphate (S1P) [6]. SphK1 is widely distributed and expressed at high levels in the brain, heart, lung, and spleen tissues. The SphK1/S1P signaling pathway involves a variety of pathophysiological reactions and participates in the occurrence and development of various diseases such as tumors, autoimmunity, and inflammatory diseases [7]. The absence of SphK1/S1P can reduce the level of endoplasmic reticulum stress in cells [8]. In addition, SphK1/S1P was found to mediate the inhibitory effect of resveratrol on lung tissue remodeling [9]. In cerebral ischemia-reperfusion injury, SphK1/S1P was found to aggravate the injury by inducing endoplasmic reticulum stress and activating the NF-*κ*B signaling pathway [10]. However, there were few studies on the effect of SphK1/S1P on MI.

Therefore, in this study, Sprague-Dawley (SD) rats were used to make MI models and were treated with SphK1 inhibitor PF543 to investigate the effect of SphK1/S1P on MI. This is the first study show that SphK1 and S1P were highly expressed in rat myocardium after MI and investigated the effects of the SphK1/S1P signaling pathway on myocardial fibrosis and inflammation after MI through the use of SphK1 inhibitors. This study will bring up light on the patients with MI and give a reminder novel method to treat this disease.

## 2. Materials and Methods

### 2.1. Animals and MI Model

This study was approved by the Animal Ethics Committee of Nanjing Medical University Animal Center. A total of 80 five-to-seven-week-old male SD rats (8 weeks old, 180 ± 20 g) were used in this study. All rats were housed in the Nanjing Medical University Laboratory Animal Center and fed with clean food and water. Before making the MI model, the rat were anesthetized with 2% sodium pentobarbital (40 mg/kg). Then, the rats were placed on the operating table and removed the fur from the rat's chest. A small animal ventilator (CWE SAR-830, Orange, CA, USA) was used to maintain the rat's breathing and set the ventilator's parameters to be the tidal volume of 1 mL, the breathing rate of 110 times/min, and the breathing ratio of 1 : 1. Then, an electrocardiograph were used to detect the electrocardiogram of the rats. After cutting the skin of the rat's left chest, the rat's ribs were cut and exposed the heart. Then, the pericardium were removed and ligated the left anterior descending coronary artery with a suture. The elevation of the ST segment of the electrocardiogram indicated that myocardial ischemia occurred in the rat. Then, the left chest of the rat were sutured and continued to feed the rat for 1 day, 7 days, and 14 days. The chest cavity of the rats in the sham group were only opened without ligating the coronary arteries. The rats in the MI+PF543 (5 mg/kg) group and MI+PF543 (20 mg/kg) group were treated with PF543 (Selleck, Shanghai, China) daily subcutaneously [11, 12].

RETRACTED

### 2.2. Cardiac Function Test

After ligating the coronary arteries for 1, 7, and 14 days, we performed echocardiography on the four groups of rats to assess their cardiac function of the rats. We used a 15 MHz probe (VisualSonics Vevo 2100, Toronto, Canada) to detect left ventricular ejection fraction (LVEF), left ventricular shortening fraction (LVFS), and early diastolic mitral valve maximum velocity/atrial systole maximum velocity of mitral valve (E/A) ratio based on the results of M-mode ultrasound.

### 2.3. 2,3,5-Triphenyltetrazolium Chloride (TTC) Staining

We collected rat hearts and placed them in a -20°C refrigerator for 20 minutes. Then, we cut myocardial tissue into slices of 2 mm thickness and soaked them in 1% TTC staining solution (Sigma-Aldrich, St. Louis, MO, USA) for 20 minutes. Infarcted myocardial tissue is pale, and normal myocardial tissue is red.

### 2.4. Histological Staining

Rat hearts were collected, and myocardial tissue was washed with normal saline. Then, we used 4% paraformaldehyde to fix myocardial tissue. We used gradient alcohol for dehydration and embed myocardial tissue in paraffin. Then, we used a microtome to make paraffin blocks into paraffin sections. Before hematoxylin-eosin (HE) staining, we put paraffin slices in xylene and gradient alcohol for dewaxing and hydration. Then, we stained the cell nucleus with hematoxylin solution (Beyotime, Shanghai, China) for 1 minute. After rinsing slices with running water, we used 1% hydrochloric acid alcohol for differentiation. Then, we used eosin solution (Beyotime, Shanghai, China) to stain the cytoplasm. Finally, we used neutral gum for sealing. In addition, we used Masson trichrome staining kit (Beyotime, Shanghai, China) for staining according to the manufacturer's instructions. Collagen fibers appear blue and muscles appear red.

RETRACTED

### 2.5. Immunohistochemical (IHC) Staining

After dewaxing and hydration using xylene and gradient alcohol, we placed the slices in citrate buffer and heated them to 95°C for 20 minutes. Then, we used 3% H_2_O_2_ to incubate myocardial tissue for 30 minutes. 10% goat serum was used to block myocardial tissue for 1 hour. Then, we used primary antibody dilution (SphK1, ab61148; S1P, ab224618; *α*-SMA, ab5694; collagen I, ab34710, Abcam, Cambridge, MA, USA) to incubate myocardial tissue at 4°C overnight. After washing the slices with phosphate buffer solution (PBS), we used secondary antibody dilution (GeneTech, Shanghai, China) to incubate myocardial tissue at room temperature for 1 hour. Then, we used diaminobenzidine (DAB) developer (GeneTech, Shanghai, China) for color development. Finally, we stained the cell nucleus with hematoxylin solution and sealed slices with neutral gum.

### 2.6. Enzyme-Linked Immunosorbent Assay (ELISA)

After collecting the rat serum, we detected the concentration of interleukin- (IL-) 1*β*, IL-6, and tumor necrosis factor (TNF)-*α* in the rat serum by ELISA kits (R&D Systems, Emeryville, CA, USA). We added samples and standards to 96-well plates and incubated them with a working solution according to the manufacturer's instructions. After stopping the reaction with the stop solution, we used a microplate reader (Molecular Devices, San Jose, CA, USA) to detect the absorbance of each well at 450 nm. Finally, we draw a standard curve according to the standard and calculated the concentration of the sample.

### 2.7. Cell Culture

The rat myocardial cell line (H9c2) used in this study was obtained from the National Institutes of Health. We used Dulbecco's Modified Eagle's Medium (Gibco, Rockville, MD, USA) containing 10% fetal bovine serum (Gibco, Rockville, MD, USA) and 1% penicillin plus streptomycin (Gibco, Rockville, MD, USA) to culture H9c2 cells. H_2_O_2_ was used to induce H9c2 cell injury.

### 2.8. RNA Isolation and Quantitative Real-Time Reverse Transcription-Polymerase Chain Reaction (RT-PCR)

We used TRIzol (Invitrogen, Carlsbad, CA, USA) to extract RNA from myocardial tissue and H9c2 cells. A spectrophotometer was used to detect the concentration of RNA. We then used reverse transcription kits (Vazyme, Nanjing, China) to reverse mRNA to complementary deoxyribose nucleic acid (cDNA). We used SYBR Green PCR Master Mix (Vazyme, Nanjing, China) to perform quantitative PCR on cDNA. Glyceraldehyde 3-phosphate dehydrogenase (GAPDH) was used as an internal reference to calculate the relative expression of different indicators. 2^-*ΔΔ*Ct^ was used to represent the relative expression of different indicators. Primers for RT-PCR was shown in Table 1.

RETRACTED

### 2.9. Cell Counting Kit-8 (CCK8) Assay

We seeded H9c2 cells into 96-well plates and treated them with H_2_O_2_ and PF543. Then, we added 10 *μ*L of CCK8 reagent (Dojindo Molecular Technologies, Kumamoto, Japan) to each well. After incubating the cells in an incubator for 2 hours, we used a microplate reader to detect the absorbance of each well at 450 nm in the dark.

### 2.10. Immunofluorescence (IF) Staining

We put cell slides in the 24-well plate and seeded the cells on the slides. After treating the cells, we discarded the medium and washed the cells with PBS. Then, we treated H9c2 cells with 4% paraformaldehyde and 0.01% Triton X-100 in sequence. After blocking the cells with 10% goat serum, primary antibody dilution were used (caspase3, ab13847; caspase9, ab32539, Abcam, Cambridge, MA, USA) to incubate the cells overnight at 4°C. Then, we used secondary antibody dilution (Abcam, Cambridge, MA, USA) to incubate the cells in the dark for 1 hour and stained the cell nucleus with DAPI. Finally, we used a fluorescence microscope to observe the staining results.

### 2.11. Statistical Analysis

Statistical Product and Service Solutions (SPSS) 21.0 (IBM Corp., Armonk, NY, USA) were used to analyze the data in this study. The mean ± standard deviation was used to represent the measurement data. We analyzed pairwise comparisons by *t*-test, and we used analysis of variance to analyze differences between multiple groups. *p* < 0.05 indicated that the difference was statistically significant. All experiments were repeated three times.

## 3. Results

### 3.1. SphK1 Was Highly Expressed in Rat Myocardium after MI

At 1 day, 7 days, and 14 days after constructing the MI model, we detected the MI area of rats by TTC staining. The results showed that the MI area of rats was larger than that of the sham group and the MI area of rats was the largest after 14 days of modeling (Figure 1(a)). The results of cardiac function tests showed that after ligating the coronary arteries, the cardiac function of the rats decreased significantly (Figures 1(b)–1(d)). We detected the structural changes of rat myocardium by HE staining (Figure 1(e)) and Masson trichrome staining (Figure 1(f)). Myocardial cells of MI rats were disorderly arranged, and there was a large accumulation of collagen in the interstitium. These results indicated that the MI rat model was successfully established. The results of IHC staining (Figure 1(g)) and RT-PCR (Figures 1(h), and 1(i)) showed that the expressions of SphK1 and S1P were increased in the myocardium of rats after MI.

RETRACTED

### 3.2. PF543 Reduced Myocardial Fibrosis in Rats after MI

The previous results found that at 7 days after MI, the myocardial tissue of the rat has already suffered evident injury and fibrosis, so we chose the 7-day modeling time for follow-up experiments. Considering SphK1 was highly expressed in rat myocardium after MI, we used SphK1 inhibitors to inhibit SphK1 activity and detect changes in rat myocardial structure. The results of HE staining (Figure 2(a)) and Masson trichrome staining (Figure 2(b)) showed that after treatment with PF543, the structure of rat myocardial tissue was significantly improved and collagen was reduced. IHC staining detected the expression of *α*-smooth muscle actin (*α*-SMA) and collagen I. After MI, the expression of *α*-SMA and collagen I in the myocardium of rats was significantly increased while PF543 decreased their expression (Figure 2(c)).

### 3.3. PF543 Improved Cardiac Function and Inhibited Inflammation in Rats after MI

We detected the changes in inflammatory factors in rat serum by ELISA (Figure 3(a)). The expression of IL-1*β*, IL-6, and TNF-*α* in the serum of MI rats increased significantly, while PF543 inhibitor of Sphk1 reduced the expression of these inflammatory factors and a high concentration of PF543 had better effects. RT-PCR results also found that PF543 can reduce the RNA levels of these inflammatory factors, IL-1*β*, IL-6, and TNF-*α* (Figure 3(b)). The results of TTC staining showed that PF543 can reduce the MI area (Figure 3(c)). The results of cardiac function tests showed that PF543 improved the cardiac function of rats, which was manifested by the increase of LVEF (Figure 3(d)), LVFS (Figure 3(e)), and E/A (Figure 3(f)).

### 3.4. PF543 Improved the Viability of H9c2 Cells and Inhibited Their Apoptosis

To determine the role of SphK1 in myocardial cells, we used SphK1 inhibitor PF543 to stimulate H9c2 cells. We detected the effect of different concentrations of H_2_O_2_ and PF543 on the proliferation ability of H9c2 cells through the CCK8 assay. 500, 700, and 1000 *μ*M of H_2_O_2_ were found to significantly reduce the proliferation ability of H_2_O_2_ cells, so we used 700 *μ*M H_2_O_2_ to induce H9c2 cell injury (Figure 4(a)). In H9c2 cells treated with PF543, the best results were obtained with 10 *μ*M PF543 (Figure 4(b)). In addition, stimulation of PF543 improved H_2_O_2_-induced cell injury (Figure 4(c)). IF staining detected the expression of apoptosis-related molecule caspase3/9. The expression of caspase3/9 in H9c2 cells induced by H_2_O_2_ was significantly higher than that in the control group, while the stimulation of PF543 reduced the expression of caspase3/9 (Figures 4(d) and 4(e)). RT-PCR results also showed that inhibition of SphK1 can reduce the expression of caspase3/9 and Bax in H9c2 cells and can increase the expression of anti-apoptotic molecule Bcl2 (Figure 4(f)).

RETRACTED

## 4. Discussion

MI is one of the primary causes of human death and the pathophysiological mechanism of myocardial injury after MI has been a hot research topic in the field of cardiovascular disease [1]. Several pathophysiological mechanisms explain the occurrence and development of myocardial injury after myocardial infarction. Braunersreuther et al. [13] demonstrated the role of oxidative stress in promoting myocardial injury after MI using a mouse model of myocardial injury. Zhou et al. [14] found excessive inflammation in patients after MI in many clinical studies. Khalilzadeh et al. [15] also explained the progression of myocardial injury after MI in a rat model with cell calcium overload. This study found that the expressions of SphK1 and S1P in the myocardium of rats after MI increased significantly with the time of MI, indicating that SphK1/S1P was involved in the disease process of MI. After treating MI rats with PF543, the myocardial structure of the rats was significantly improved and the degree of fibrosis was reduced. The inflammation level of MI rats also decreased with the treatment of PF543. In addition, PF543 was also found to promote the proliferation of H9c2 cells *in vitro* and reduce H_2_O_2_-induced apoptosis. Therefore, SphK1/S1P may be a potential therapeutic target for MI.

Myocardial fibrosis is an important cause of long-term poor prognosis in MI patients and compensatory response to myocardial injury [2]. The occurrence and development of many cardiovascular diseases are related to myocardial fibrosis, which is characterized by the accumulation of activated cardiac fibroblasts (myofibroblasts) and excessive deposition of extracellular matrix [16, 17]. Myofibroblasts are fibroblast-like cells that can express *α*-SMA. They have both the contraction function of smooth muscle cells and the function of fibroblasts to secrete extracellular matrix [18]. Unbalanced collagen ratio, disordered arrangement, or abnormal concentration will promote myocardial fibrosis, increase the stiffness of the ventricular wall, and reduce the compliance of the ventricular wall, resulting in the weakening of myocardial diastolic function and cardiac diastolic dysfunction [19]. The SphK1/S1P signaling pathway has been studied in detail in fibrotic diseases. Xiu et al. [20] found that stimulation of bleomycin or TGF-*β* can lead to increased levels of SphK1 and S1P in lung tissue and human embryonic lung fibroblasts (HELF), respectively. Sferra et al. [21] also found in bleomycin-induced lung fibrosis model mice that the expression of SphK1 mRNA and protein in the lung tissue of mice increased. After the SphK inhibitor was used, the degree of bleomycin-induced lung injury and fibrosis was significantly reduced. At the same time, in HELF stimulated by bleomycin or TGF-*β*, the expression of SphK1 mRNA and protein increased, and the expression of fibrosis phenotype-related markers fibronectin and *α*-SMA also increased. Bleomycin-induced lung injury and fibrosis were significantly reduced when SphK inhibitor was used. These results indicated that the pulmonary fibrosis process mediated by TGF-*β* may rely on SphK1 as the rate-limiting enzyme for the synthesis of S1P. In addition, the intracellular SphK1/SIP signal was also found to result in increased collagen expression of fibroblasts in the liver [22]. Therefore, we investigated the effect of SphK1/S1P signaling pathway on myocardial fibrosis in MI. The results of Masson trichrome staining and IHC staining showed that myocardial tissues of rats had obvious fibrosis at 7 and 14 days after MI, while the treatment of PF543 (inhibitor of Sphk1) reduced the degree of myocardial fibrosis.

RETRACTED

SphK1 and S1P are an important class of signaling molecules with important biological activities. They are involved in the regulation of cell growth, differentiation, senescence, and death [23]. After S1P acts on the S1P receptor (S1PR), it can play an important regulatory role in many physiological and biochemical processes. In myocardial tissue, S1P can regulate cardiac electrophysiology and contractile activity, and S1PR1 can inhibit cAMP-mediated L-type calcium ion channels in myocardial cells, reducing myocardial contractility [24]. G protein-gated inward rectifier potassium channels in myocardial cells can be activated by S1PR3, reducing myocardial contractility [25]. In this study, the use of SphK1 inhibitors effectively increased the LVEF, LVFS, and E/A of MI rats, so inhibition of SphK1/S1P may become one of the methods to improve the cardiac function of MI rats. In addition, some studies have shown that when inflammation occurs in the body, the expression of SphK1/S1P signaling pathway in cells at the site of inflammation is significantly increased [26, 27]. SphK1 and S1P were found to be significantly increased in the spinal cord of patients with multiple sclerosis and the serum and cerebrospinal fluid of mice with autoimmune encephalomyelitis [28]. These indicated that the SphK1/S1P signaling pathway may be involved in the progression of inflammatory diseases [29, 30]. We found that the expression of inflammatory factors in MI rats increased significantly, and PF543 showed a good anti-inflammatory effect.

RETRACTED

To our knowledge, this is the first study to investigate the effect of the SphK1/S1P signaling pathway on MI and previous studies did not report. Our results suggested that SphK1/S1P inhibitor has a good application prospect for MI. However, this study did not contain the clinical tissues in patients, which lack the verification of the results. Besides, the underlying mechanism of this study is not clarified, which needs further studies to verify it. Next, we can focus on how the SphK1/S1P relieve MI and which molecule plays a main role in the progress.

## 5. Conclusions

To sum up, this is the first study to show that SphK1 and S1P were highly expressed in the rat myocardium after MI and investigated the effects of the SphK1/S1P signaling pathway on myocardial fibrosis and inflammation after MI through the use of SphK1 inhibitors. The SphK1/S1P signaling pathway may become a new target for clinical treatment of MI.

## Figures and Tables

**Figure 1:** SphK1 was highly expressed in rat myocardium after MI. (a) Myocardial ischemic area of rats was increased from 1to 14 days. (b–d) LVEF, LVFS, and E/A of rats decreased from 1 to 14 days. (e, f) HE staining and Masson trichrome staining of rat myocardium (200x). (g) IHC staining results showed that the expression of SphK1 and S1P in rat myocardium (200x) increased from 1 to 14 days. (h, i) mRNA expression of SphK1 and S1P in rat myocardium increased from 1 to 14 days. (“^∗^” means *p* < 0.05 vs. the sham group), based on Student's *t*-test. Scale bar: 50 *μ*m.

**Figure 2:** PF543 reduced myocardial fibrosis in rats after MI. (a, b) HE staining and Masson trichrome staining of rat myocardium (200x). (c) IHC staining results of *α*-SMA and collagen I in rat myocardium (200x). Bar: 50 *μ*m.

**Figure 3:** PF543 improved cardiac function and inhibited inflammation in rats after MI. (a) ELISA results of IL-1*β*, IL-6, and TNF-*α* in rat serum. (b) mRNA expression of IL-1*β*, IL-6, and TNF-*α* in rat myocardium. (c) Myocardial ischemic area of rats. (d–f) LVEF, LVFS, and E/A of rats. (“^∗^” means *p* < 0.05 vs. the sham group; “^#^” means *p* < 0.05 vs. the MI group), based on Student's *t*-test.

**Figure 4:** PF543 improved the viability of H9c2 cells and inhibited their apoptosis. (a, b) CCK8 assay results of H9c2 cells on H_2_O_2_ and PF543. (c) CCK8 assay results of H9c2 cells in four groups. (d, e) IF staining results of caspase3/9 in H9c2 cells (200x). (f) mRNA expression of caspase3/9, Bax, and Bcl2 in H9c2 cells. (“^∗^” means *p* < 0.05 vs. the control group; “^#^” means *p* < 0.05 vs. the H_2_O_2_ group), based on Student's *t*-test.

RETRACTED

**Table 1:** RT-PCR primer sequences.

Name	Sense/antisense (S/AS)	Sequences (5′-3′)
SphK1	S	TCCACCCGGAGAGAACA
	AS	CCCCTCCAGCCTCAAAC
S1P	S	TGTGGCTGGCTTAGTGTG
	AS	AGGCTCTGTGTCTTTGGTG
caspase3	S	TGGACAACAACGAAACCTC
	AS	ACACAAGCCCATTTCAGG
caspase9	S	GGAGTTGACTGAGGTGGGA
	AS	AGCAAGGAAGACACTGGGA
Bax	S	CGGCTGCTTGTCTGGAT
	AS	TGGTGAGTGAGGCAGTGAG
Bcl2	S	GTCACAGAGGGGCTACGA
	AS	GTCCGGTTGCTCTCAGG
GAPDH	S	GTTGTGGCTCTGACATGCT
	AS	CCCAGGATGCCCTTTAGT

## Data Availability

The data could be obtained from contacting the corresponding author.
